The article "Green R & D investment, ESG reporting, and corporate green innovation performance" was retracted in 2025. Reasons: concerns about the results or conclusions; concerns about the peer review; concerns about the authorship.

# Green R & D investment, ESG reporting, and corporate green innovation performance

**DOI:** 10.1371/journal.pone.0299707

**Published:** 2024-03-28

**Authors:** Fawad Rauf, Wang Wanqiu, Khwaja Naveed, Yanqiu Zhang

**Affiliations:** 1 College of Economics and Management, Beijing University of Technology, Beijing, China; 2 Department of Accounting, College of Business and Economics, United Arab Emirates University, Al Ain, Abu Dhabi; 3 Management College, Beijing Union University, Beijing, China; Universidad Internacional de La Rioja, SPAIN

## Abstract

Given the contradictory empirical evidence on the relationship between green R&D expenditure and corporate Green Innovation performance (GIP), The present research study is a distinctive investigation into the moderating impacts of ESG reporting on this relationship. We utilized a data collection of 3,846, firm-year observations of A-share listed firms in China from 2016 to 2022 from CSMAR and Bloomberg databases. The firm’s Corporate GIP is assessed and measured by looking at the total quantity of green patents. Lastly, models with multiple regression analyses and fixed effects were employed. The findings show that ESG reporting has a positive and significant impact on the association between corporate GIP and green R&D expenditure, implying its compensating and supportive function in the form of green signals in green outputs. This research could help executives and lawmakers, especially in developing countries to build innovative environmental strategies for business sustainability.

## 1. Introduction

Companies should look for current possibilities to improve their situation and market position in comparison to competitors in today’s market rivalry [1]. Earnings and competitive advantage are earned through innovation [2, 3]. and a concomitant desire to achieve economic stability and environmental leadership [4, 5]. On either side, innovation is frequently risky and costly. As a result, the key question is whether advanced innovation that promotes financial efficiency can simultaneously reduce environmental damage. Greening, innovation, teamwork, openness, and social inclusion are the five main development ideas in China’s new phase.

China’s economic growth and development rests heavily on the individual performance of its companies [6]. However, despite being the world’s second-largest economy, China’s Environmental Performance Index (EPI) ranking of 120th out of 180 countries (Yale University, Columbia University, & World Economic Forum, 2018) indicates significant environmental challenges [7]. As the global trend towards sustainable business practices gains momentum, Chinese companies must embrace Corporate Green Innovation Performance (CGIP) to improve their financial and environmental performance simultaneously [8, 9]. This involves integrating environmental responsibility into innovative activities to minimize negative environmental impacts. Notably, the "One Belt, One Road" initiative, while promoting economic progress, has also led to increased energy consumption and carbon emissions in many participating countries [10]. Therefore, green investment within this initiative becomes crucial to achieve a win-win scenario for society, the environment, and national finances.

While a narrower information gap between corporations and shareholders might initially appear detrimental, studies have shown it can lead to positive outcomes. The decreased information gap between corporations and their shareholders has resulted in a decrease in the value of firm assets and growth in the firm’s value [11, 12]. This implies that increased transparency allows companies to focus on long-term value creation for all stakeholders, rather than short-term gains through information manipulation [13, 14]. One key tool in fostering this transparency is environmental, social, and governance (ESG) reporting. In 2008, ESG certificates started to be issued under ISO 9000 and ISO 14001, whereby most large corporations have increasingly adopted compliance in their annual reports to openly publish their ESG activity [15, 16]. Murphy [17] suggest three plausible causes behind this trend: a desire to fulfill societal expectations of corporate responsibility, enhance legitimacy, and encourage investment in green R&D. Ultimately, active engagement with ESG principles and transparent reporting can benefit corporations in two ways. Firstly, it can create a positive public image, presenting the company as dignified and ethical. Secondly, it helps meet stakeholder expectations and build trust, leading to better long-term performance [18–22]. The well-known Berle’s-Dodd debate has piqued the public’s interest in CSR. Berle’s [23] According to others, companies should only be examined if they raise the worth of their shareholders. Dodd’s [24] viewpoint advocates the idea that corporations should be held responsible to investors and ordinary individuals. ESG typically includes obligations to employees, lenders, consumers, social welfare, the environment, and profit. In other words, ESG is the commitment to stakeholders rather than simply investors. By focusing on firms’ responsibilities to shareholders, it has been discovered that ESG and firm performance are linked [25–29]. As a result, it is necessary to examine the effect of ESG reporting on green R&D investment as well as the moderation function of ESG reporting on corporate GIP.

While existing research points to a direct link between corporate green innovation performance (GIP) and green R&D, the nature of this relationship remains complex. Past studies have explored various outcomes, ranging from positive to negative to neutral, when examining the impact of green R&D on GIP [30]. This suggests that additional factors beyond the simple correlation may be at play, potentially influencing the observed connections. Li et al. [31], and Pham & Tran [32] highlight the possibility of such intervening variables, urging further investigation into their role in shaping the relationship between green R&D and GIP.

A growing emphasis has been placed on the valuable effects of ESG reporting on an enterprise’s financial capability [33, 34]. Financial execution can be examined and evaluated throughout time by shareholders, management, and other investors using ESG ratings and reports [35–37]. There are three plausible reasons why ESG was chosen as the research variable in this study. First, ESG information can effectively illustrate a company’s financial efforts in ESG [38, 39]. Secondly, ESG data is the most impartial way to evaluate the long-term performance of a firm, indicating valid differentiation in the model. Lastly, extant research on ESG reporting has reawakened attention. ESG reporting combines sustainability data, ESG, and sustainable [40, 41]. In developing countries, the association between ESG reporting and research is less widespread [42, 43], Furthermore, the correlation between ESG and corporate GIP is still poorly understood. As a result, the goal of this research is to identify how ESG reporting influence the relationship between green R&D investment and corporate GIP, As China’s economic development places a larger emphasis on social and environmental issues, ESG practices are projected to become more popular. The findings of that probe will add to our understanding of green initiatives in developed economies.

Sustainability and social responsibility theories form the backbone for analyzing the links between corporate GIP, ESG reporting, and investments in green R&D [44, 45]. Sustainability theory advocates for businesses to factor in economic efficiency, social accountability, and environmental preservation during their operations [44, 46]. A company’s performance serves as a yardstick to assess its effectiveness across these three realms. Strong corporate performance signals profitability, growth, and a greater inclination towards prioritizing social responsibility and environmental sustainability [47]. Moreover, a company’s commitment to sustainability and social responsibility is underscored by its investment in green R&D, a practice closely aligned with the concept of social responsibility [44, 48].

This research will contribute to the corpus of existing information in the following ways: firstly, the vast majority of current ESG research focuses on the relationship between ESG reporting and financial success; however, the association between ESG reporting and corporate GIP has yet to be discovered. We’re trying to fill a gap in the ESG literature. Secondly, this study adds to the current body of information by looking into the link between green R&D investment, ESG reporting data and corporation GIP While socially responsible investing has a huge context in the Chinese scenario, it is less studied in the scenario of rising markets in industrialized countries. Our findings could lead to new approaches to increasing corporate GIP through R&D investment and ESG reporting.

Finally, for executives observing the development of ecological policies for innovation, this study expands on our understanding of the corporate GIP mechanisms that underlie the observed relationship between green R&D investment, ESG reporting, and corporate GIP. They proposed the overinvestment hypothesis in this setting using agency theory. It implies that the benefits of green R&D investments in enhanced family businesses stem from ESG reporting. To the utmost of our abilities, no previous published study has discovered that ESG reporting influences the connection that exists between green R&D investment and company GIP.

The following structure depicts the paper’s structure. The framework for the literature and the creation of hypotheses are offered in Section 2. The technique, sample, details, empirical frameworks, and sample are all provided. in Section 3. Section 4 examines empirical results. The closing, implications, limitations, and future direction are presented in Section 5.

## 2. Development of a theoretical framework and hypotheses

To fill these gaps in research, a comprehensive model has been created using agency theory, resource-based view (RBV) theory, and legitimacy theory. Agency theory highlights the potential for conflict between shareholders and other stakeholders, creating an obstacle to effective ESG reporting. To manage this, Cormier et al. [49] suggest that companies often utilize different information reports to portray varying levels of firm performance to different stakeholder groups. This raises the question of how reliable ESG reporting is. Traditionally, research on ESG reporting focused on its role in enhancing a company’s legitimacy rather than directly investigating its motivations. For example, Mayer & Ducsai [50] found that emphasizing tax benefits and minimizing information asymmetry are seen as key benefits of ESG reporting for enhancing a company’s image of responsible conduct.

In terms of legitimacy theory, According to several experts, the perception of ESG reporting is primarily dependent on this hypothetical structure [51]. According to this theory, Firms act as objects when they accept achievements that are constrained by social norms, expectations, and standards [52, 53]. Van Staden and Hooks [54] suggested that businesses adopt reactive or proactive tactics to get credibility. The reactive techniques refer to ESG information provided by businesses in response to unfavorable or major occurrences. For years, the company’s strategy for delaying the rise in legality issues has been utilized to put legitimacy ideas to the test [55–57]. Birkey et al. [58], evaluated whether or not there is a significant relationship between the corporate sector and the importance of ESG reporting [59]. Other researchers contended that when compared to enterprises in ecologically sensitive industries, Companies in environmentally sensitive areas publish more ESG reporting data, which also demonstrates the study’s effectiveness [60]. Hoffman [61]was concerned that businesses in similar regions and states would isolate the many parties involved in their methods, providing a receptive environment in which to evaluate one another to achieve public attention and validate performance [61]. Similarly, Gray et al. [62], recommended linking disclosure policies to business and government power, underlining the legality theory’s persistence [62]. In addition, Castello and Lozano [63] anticipated that there would be a demand for the Dow Jones Sustainability Index (DJSI) as a moral legality model. As a result, participation in DJSI is critical because it makes people recognize that the organization’s performance fulfills public expectations, which can be a strong indicator of its legitimacy [64]. According to Campbell [65], companies can use non-financial information to respect societal values and beliefs while also acting environmentally responsible, according to research suggestions [66].

The Resource-Based View (RBV)states, Resources and managerial abilities are critical in gaining a competitive advantage [67]. In addition, it asserts that firms can expand over time and gain a competitive advantage by addressing typical environment-related problems. Hart [68] remarked regarding the shortcomings of RBV theory that it does not consider any contact between the natural administrative environment and the association itself. This elimination was used to make sense, However, it is obvious that the environment plays an important role in developing a competitive advantage [68]. Natural resources as well as skills, according to Hart and Dowell [69], calculate the economics of pollution reduction. Environmental resources, avoidance of pollution strategies, and managerial qualities all contribute to long-term success [69]. By emphasizing the social, economic, and environmental components of ESG, Researchers can use RBV’s natural theory to quantify the performance of companies [70]. This research complements its framework for ESG reporting (economic, social, and environmental assessment), corporate GIP, and company performance via the lens of natural RBV theory.

### 2.1. Green (R & D) investment and corporate GIP

When evaluating a company’s Green Innovation Performance (GIP), it’s crucial to highlight the pivotal role played by investment in green Research and Development (R&D) activities [30, 71, 72]. It’s widely acknowledged as a critical factor in bolstering both economic advancement and the value of businesses [73]. Creating novel and inventive products while attaining expertise and proficiency in comprehending intricate processes [74], and acquiring innovation is crucial. Elevated levels of investment in green R&D can significantly facilitate the establishment and execution of Green Innovation Performance (GIP). Developing accessible technology can notably influence the company’s growth in productivity [75, 76].

According to the Natural Resource-Based View (RBV) perspective, businesses should integrate environmental sustainability into their planning processes, thereby contributing to the development of innovative strategies [68]. Consequently, this framework emerges as a means to fortify the company’s capacity to navigate uncertainty and cultivate invaluable managerial expertise [77]. This plays a pivotal role in the company’s capability to conduct green innovation performance (GIP) activities and expand its GIP resources [78]. Salter & Laursen (2006) highlighted the importance for businesses to possess environmental resources in order to foster innovation [79]. Triguero, Mondejar, Moreno, and Davia [80] recognize that having superior access to external data heightens the potential for growth in GIP [80, 81], Elevated green investment in research and development can assist enterprises in acquiring these resources. The rapidly changing technological landscape of today not only encourages innovation but also surpasses the innovation pace seen in the past [82]. The company needs innovative strategies to swiftly adapt to unforeseen changes and to provide diverse solutions that address latent consumer needs [83, 84]. Augmented investment in green Research and Development (R&D) can assist the firm in acquiring reliable market data crucial for advancing technological developments [85], and focus on a broad spectrum of highly valuable and distinctive products, along with enhanced manufacturing advancements, to enhance their overall performance [86]. Companies investing in green research and development tend to face reduced risks of obsolescence [87]. They achieve this by enhancing their technological resources and expertise while remaining mindful of current advancements in technology [88], while also acknowledging emerging trends in this context [79].

Pollution avoidance empowers companies to cease polluting manufacturing processes, modify construction methods to reduce life cycle outcomes, and develop new products with reduced life cycle impacts [68]. Reducing business expenses is a potential outcome. A sustainable environment can also support the development of organizational skills within companies [89, 90]. Companies can benefit from reduced cost factors, load management, recycling initiatives, and maintenance strategies, among other aspects of product creation [91, 92]. To cut down on operational expenses, it’s important to note that eliminating pollution could potentially elevate demand for a company’s products among environmentally conscious consumers. Globally, environmentally conscious businesses are increasingly preferred due to their sustainable practices, cost reductions, and increased endorsements [93]. Stronger support can incentivize environmentally conscious enterprises to leverage their management practices as selling points, distinguishing themselves from competitors. Consequently, green organizations are demonstrating a growing array of technological breakthroughs in the market [94]. It’s considered among the most assertive approaches to leverage environmental progress for aiding firms in enhancing their management capabilities. This allows them to employ more adaptable strategies across various scenarios and address societal concerns effectively [95]. We believe that Corporate (GIP can aid firms in enhancing their products and internal processes while reducing operational costs. Additionally, it can lower overall risk by differentiating them from competitors and bolstering their external reputation and trustworthiness [77].

Certain companies have pioneered novel methodologies, resulting in increased investment in green R&D. As the company’s commitment to green R&D expands, leaders can achieve more efficient GIP by leveraging resources, capabilities, and ingenuity. This involves empowering employees, refining processes, and adopting cutting-edge technologies. They would be satisfied with an elevated GIP both internally and externally, achieving more with fewer resources and yielding a superior overall return on investment [96]. As a result, boosting green R&D investment provides a long-term and operational benefit for GIP.

**Hypothesis (H1):** Green R&D investment correlates positively with corporate GIP.

### 2.2. Corporate GIP and ESG reporting

GIP is multifaceted and cannot be encapsulated by a singular term [97], This is often regarded as the intersection of technological advancement and environmental effectiveness [98]. The advancements highlighted in this study can serve as a catalyst for progress, contributing to energy efficiency, pollution prevention, emission reduction, and overall environmental preservation. These breakthroughs in green technology support the ecological stability of natural resources. The visibility of green initiatives by firms could be influenced by Corporate GIP, impacting the number of observable implementations by these companies. Hence, in this analysis, recent claims related to green initiatives are used as a proxy variable for corporate GIP, supported by research [99, 100]. Acquiring green patents involves securing intellectual property rights for environmentally friendly innovations, technologies, or processes that contribute to sustainability and ecological preservation.

GIP significantly contributes to the economic development of manufacturing-driven nations. However, the predominant focus has traditionally centered on innovation, placing Chinese firms primarily in the innovation stage rather than prioritizing green growth [101]. Uniting financial progress with green development can create new avenues for a resilient economy. Technological advancements have become a critical factor enabling green growth. However, continuously driving technological advancements to facilitate green development can be quite costly [102, 103]. The dynamic cultivation of corporate green innovation performance (GIP) and the acceleration of green transformation hinge on whether the evolution towards green initiatives can generate environmental advantages for firms while balancing increased economic benefits and heightened corporate significance.

ESG reporting holds significant weight in non-financial information disclosure. In China, organizations have initiated the publication of their ESG reports, unveiling corporate performance metrics and outlining commitments towards ESG principles [104]. Through excellent oversight of ESG implementation by all stakeholders, ESG is ascribed to achieving maximum social prosperity and sustainability [105]. Diminished environmental impacts and heightened ESG reporting practices are widely acknowledged and embraced across multiple countries [106]. In January 2008, the State Council’s Resources Management Committee and the State-owned Assets Supervision and Administration Commission (SASAC) released guidelines for social responsibility information reports by parent companies, spurring enthusiasm among governing companies to issue ESG reports. Notably, statistics from SASAC indicate active ESG report publication by major corporations. In 2014 and 2015, approximately 57.55% and 75.89% of central enterprises, respectively, tended to release ESG reports [107]. Between 1998 and 2015, China’s overall societal investment in Research and Development (R&D) within the GDP surged from 0.69% to 2.1%. The total social investment in 2015 reached 1430 billion RMB, with green R&D investment constituting over 77% of GDP and audit accounting for 2.10% of GDP. Regarding distribution, R&D investments in Chinese companies, state-owned research facilities, and universities in 2015 were 76.8%, 15.1%, and 7%, respectively. The following hypothesis is therefore put forward:

**Hypothesis (H2):** *There is a significant association between corporate GIP and ESG reporting*.

### 2.3. Moderating role of ESG reporting on corporate GIP—Green R&D investment

Green research and development (R&D) investment plays a crucial role in a company’s success. It not only fosters the development of technical advancements but also enhances the company’s capacity to create and disseminate innovations, especially in today’s dynamic and constantly evolving environment [108]. Green R&D investment leverages both tangible and intangible assets, such as technological resources, financial investments, and skilled R&D personnel. In this context, the Resource-Based View (RBV) can aid in understanding how to effectively utilize abundant and distinctive resources to enhance operational capabilities and introduce innovative products. This approach enables the company to cultivate sustained moderate profits while maintaining strong performance.

Excessive investment in green research and development (R&D) within a company, primarily due to inherent problems and budgetary constraints, may not necessarily bolster internal productivity. Instead, it could result in neglecting Environmental, Social, and Governance (ESG) performance. This might occur due to the insecurity of internal resources caused by inefficient R&D investment practices. Additionally, an overemphasis on R&D could lead to employee dissatisfaction, particularly stemming from a lack of consideration for environmental concerns and ESG norms [109, 110]. ESG efforts have often been viewed as costly endeavors for businesses. Consequently, corporations may perceive ESG operations as supplementary and expensive measures that negatively impact the manufacturing industry [111].

Innovative green businesses are showcasing a growing array of technological advancements within the market [94]. Leveraging environmental progress as a proactive strategy can significantly aid businesses in fortifying their management capabilities, enabling them to employ more adaptable approaches across diverse scenarios and address societal concerns effectively [95]. We believe that organizations dealing in corporate GIP can improve their goods and internal processes while lowering their operational costs, They can also reduce overall revenue by differentiating themselves from other members and improving their external reputation and reliability [77].

Porter [112] suggested that robust and fitting environmental practices would drive businesses to embrace Corporate GIP in energy conservation and environmental protection. Consequently, several scholars have concluded that environmental regulations can foster the advancement of corporate GIP [113–115]. It’s suggested that mandatory ESG reporting serves as an environmental regulatory strategy, aiming to constrain pollution releases and spur Corporate Green Innovation Performance (GIP). The idea is that once companies disclose their ESG activities, government bodies and advocacy groups can leverage technology to pressure polluting firms into reducing their emissions by publicly highlighting their environmental impact [116, 117].

In general, mandatory ESG reporting impacts company GIP in two primary ways. Firstly, ESG reporting data can mitigate agency problems, aiding managers, and shareholders in maintaining control over ownership. In instances where information inconsistency worsens the agency problem, mandatory ESG reporting, as a non-financial reporting technique, might reduce information inconsistencies and improve monitoring [118]. A professional business model states that directors can reduce the risk of innovation, and increasing supervision can increase incentives to innovate [119]. Secondly, ESG reporting information, as an environmental guideline, can encourage corporations’ GIP (see Fig 1). Hence, the following hypothesis is proposed:

**Hypothesis (H3):** *ESG reporting positively moderates the association between green R&D investment*, *and corporate GIP*.

**Fig 1:** Green R & D investment, ESG reporting, and corporate GIP.

## 3. Data collection, quantification, and study methodology

### 3.1. Sample and data

That’s an extensive dataset covering Chinese corporations listed on the Shanghai and Shenzhen stock exchanges from 2016 to 2022, with a focus on non-financial companies. The data was sourced primarily from the Chinese Stock Exchange and the Accounting Research (CSMAR) as well as the Bloomberg Database, which are reputable sources for information on Chinese-listed enterprises. The manual acquisition of ESG scores indicates a hands-on approach to assessing environmental, social, and governance aspects. Emphasizing industrial sectors aligns well with the typical involvement of firms in green Research and Development (R&D) initiatives. With 3,846 firm-year observations obtained after eliminating missing data points, your dataset seems robust and comprehensive for analysis purposes.

### 3.2. Corporate Green Innovation Performance (GIP)

In this study, corporate green innovation performance (GIP) is employed as a dependent variable, with two components: intention and performance The China National Holding Administration (CNIPA) has mixed 10137 application patents from 327 energy-intensive listed companies, such as patents, effectiveness models, etc. In addition, 2971 green patents have been erased in this research to get the keywords: 1. greenish 2. Sustainable 3. Low greenhouse gas emissions 4. Environmental 5. Clean 6. Saving energy 7. Protecting 8. Ecology 9. Waste disposal 10. Environmental protection, and 11. Emissions reduction from the 10137 evaluation patents. A tendency towards Green Innovation can be a two-variable that equals 1 if a firm acquires a minimum of one green evaluation patent and nil otherwise. In this investigation, GIP is represented by the number of green patents [120, 121].

### 3.3. Green Research and Development (R&D) investment

We adapted the items proposed by Lee and Min [122] and Cui and Wang [123] for green, Green Research and Development (R&D) investment. which reflects the organizations’ expenditure on equipment, employees, and funds. There are three factors, which are " Green R&D equipment investment makes up a sizable share of total equipment asset investment", “Employees involved in green R&D make up a sizable share of the entire workforce,” and “green capital investment R&D makes for a sizable share of total capital investment” [122, 123].

### 3.4. Moderating role of Environmental Social & Governance (ESG) reporting

We employed ESG reporting as a mediating dependent variable. To measure ESG reporting, we utilize the Social Responsibility Score provided by the Chinese ESG score company https://www.bloomberg.com/. The score is an in-depth analysis of the ESG facets of businesses with listings on the Shanghai and Shenzhen Stock Exchanges. We used an amphibious technique to create the ESG index: Recent ESG disclosure data collection has extensively employed Bloomberg’s ESG reporting [124, 125]. ESG information was evaluated utilizing the Bloomberg-published ESG reporting score of Chinese listed companies. Better ESG disclosure is indicated by a higher score. The developing method was used to evaluate the score for ESG reporting: ESG Score, $\sum_{j=1}^{11}$ × 100, where i equals 1 if the item is described and 0 otherwise and where n represents the number of items.

#### 3.2.6. Control variables

We were able to manage the issues that could have an impact on the ESG reporting in this investigation, as depicted: [126]. (1). Return on assets (ROA), is the percentage of net earnings after tax to total assets [127]; (2). firm age (FA), which was determined by the number of years from firm establishment to the inference [128]; (3). Financial Leverage (FLever) is considered a possible predictor of FP that can resolve the agency problem in a public entity. In previous studies, we calculated financial leverage using the debt-to-equity ratio [129]; (4). State-owned enterprises (SOEs) were regulated by the state or the government, and a particular factor equal to 1 was used to evaluate it [130]; (5). Tobin Q It is a variable concerning the percentage between the market value and the added value of a physical asset. (6). Chief executive officer Duality (CEOD) If the CEO also serves as the chair of the company’s board of directors, it may help to develop dependable and irrefutable governance, supporting the CEO’s consolidation of power [131]. CEO duality is a binary variable, with 1 representing ’duality’ and 0 representing ’non-duality’. (7). Firm size (FS) Firm size is taken as an indicator of FP and credibility. We measure firm size using net income (Asset) and employee number, as earlier studies had also done [132]; (8). Ownership concentration (OC) has been calculated using the total stockholding of a first key creditor [133]; (9). Investment opportunities (IO) market value of a firm multiplied by the replacement value of its assets [134]; (10). Growth opportunity (GO) is defined as the rate of increase in the company’s primary income [135]; Finally, (11). A year and Industry dummy (YI) we incorporated, we retain the year impact because of some possible threats, which are not obtained in our concepts or may occur and impact a company’s business performance industry dummies to control the particular consequence of the company [136]; All of these control variables are often used in research on Chinese firms. See Table 1.

**Table 1:** Description of variables.

Variables	Abbreviation	Measurement
Green Innovation Performance	GIP	The count of patent applications for green inventions.
Green Research & Development	R&D	The aggregate value of Research and Development (R&D) is computed by combining both Green R&D and generic R&D expenditures
Environmental Social and Governance	ESG	ESG information serves as a proxy for ESG and is quantified as a score ranging from 1 to 100. This score is assigned by a Rankins agency to a specific business each year
State Owned Enterprise	SOEs	equivalents for a dummy variable 1 if the local or regional government is the dominant owner, and 0 otherwise.
Tobin Q	Tobin Q	market value of a firm’s outstanding shares to the replacement cost of its tangible assets.
Firm Age	FA	The duration of the firm’s existence was used to establish its age.
Return of Assets	ROA	It is a factor affecting the proportion of total profits to total assets.
Financial Leverage	FLever	To determine the asset-liability ratio, divide (total liabilities) by (the total number of assets) (total resources as an average).
CEO Duality	CEOD	when an individual holds the positions of Chairman and CEO simultaneously, it is referred to as CEO duality.
Firm Size	FS	The total assets at the end of the fiscal year represent the aggregate value of all assets held by a company
Ownership Concentration	OC	Distribution of ownership stakes among shareholders in a company.
Investment Opportunities	IO	Assets that offer the potential for financial gain or return on investment
Growth opportunity	GO	characterized as the pace of expansion in a company’s main source of income.
Year and Industry	YI	In all regression analyses, Industry dummies are incorporated to manage the influences of both time (year) and specific firm characteristics.

#### 3.2.7. Empirical model

We build ordinary list square (OLS) regression models to test our hypothesis and then use fixed effect tests to investigate further.

Model 1 is used to investigate the association between green R&D investing and corporate GIP.


$${GIP}_{\left(i,t\right)}=a+\beta_{1}R\&D+\sum_{i=1}^{N}\beta_{n}{controls}_{\left(i,t\right)}+{ℇ}_{\left(i,t\right)}$$ (1)

Model (2) is used to investigate the influence of ESG Reporting on Corporate GIP:

$${GIP}_{\left(i,t\right)}=a+\beta_{2}ESG+\sum_{i=1}^{N}\beta_{n}{controls}_{\left(i,t\right)}+{ℇ}_{\left(i,t\right)}$$ (2)

Model (3) is used to investigate how ESG reporting affects the link between green R&D investment and corporate GIP.

$${GIP}_{\left(i,t\right)}=a+\beta_{3}R\&D+\beta_{4}ESG+\beta_{5}R\&DxESG+\sum_{i=1}^{N}\beta_{n}{controls}_{\left(i,t\right)}+{ℇ}_{\left(i,t\right)}$$ (3)

where i and t denote the firm and the year, respectively; b denotes the assumed parameter, and ℇ denotes the error component.

## 4. Result and discussion

### 4.1. Descriptive statistic

Table 2 displays the descriptive statistics for the important variables. The average value of GIP is 0.053. Green R&D investment and ESG reporting have mean values of 9.475, and 3.434, respectively. Furthermore, public visibility and firm transparency are significantly and positively correlated with the effectiveness of GIP, which can give us a deep understanding of our critical theoretical stance. Hence, it is evident that public visibility and firm transparency can act as moderators and companies in the context of ESG reporting and GIP, green R & D investment. The association between all explanatory factors, including control variables, is shown in Table 2.

**Table 2:** Descriptive statistics.

Variables	Mean	SD	Min	Max
GIP	0.053	0.063	0.000	1.000
R&D	9.475	2.271	4.001	21.00
ESG	3.434	0.846	1.000	8.000
SOEs	0.266	0.471	0.000	1.000
Tobin Q	1.784	1.828	0.095	32.261
FA	10.246	0.836	-18.543	42.635
ROA	10.237	4.781	1.000	56.000
FLever	0.516	0.226	0.006	1.345
CEOD	0.164	0.383	0.000	1.000
FS	0.286	0.483	0.000	1.000
OC	1.177	1.163	0.032	10.381
IO	0.158	0.372	-0.817	10.862
GO	2.443	1.951	0.746	33.684

### 4.2. Correlation matrix

Table 3 displays the correlation coefficients of the major variable’s results. The results reveal that GIP and green R&D are consistent at a 1% level, whereas ESG reporting is consistent at a 5% level. As a result, green Innovation and green R&D investment have a positive and strong relationship with mitigating ESG reporting, this also shows consistency at the 1% level among univariate affecting variables. All correlation analyses are less than 0.70, implying that the highest correlation between all variables does not rise by 0.641. As a result, no multicollinearity issue may have a significant impact on our results. The correlation coefficients of variance inflation factors (VIFs) were 0.653, suggesting that no variables were collinear.

**Table 3:** Correlations matrix.

Variables	(1)	(2)	(3)	(4)	(5)	(6)	(7)	(8)	(9)	(10)	(11)	(12)	(13)
GIP	1.000												
R&D	-0.004	1.000											
ESG	0.631**	-0.017***	1.000										
SOEs	0.042***	-0.005***	0.021***	1.000									
Tobin Q	-0.161**	0.331***	-0.156***	-0.062**	1.000								
FA	0.007***	-0.106***	0.047***	0.018**	-0.098**	1.000							
ROA	0.013***	0.561***	0.011***	0.023**	0.105**	-0.014**	1.000						
FLever	0.116***	-0.418**	0.147***	0.031**	-0.506**	0.223**	-0.102**	1.000					
CEOD	-0.134***	0.091**	-0.082**	-0.016*	0.132**	-0.001**	0.034**	-0.124**	1.000				
FS	0.047**	-0.007**	0.027**	0.491**	-0.057**	0.012**	0.017**	0.028*	-0.012**	1.000			
OC	0.097**	-0.296**	0.158**	0.015**	-0.512**	0.166**	-0.092*	0.616**	-0.124**	0.016**	1.000		
IO	-0.028**	0.166**	-0.018**	-0.001*	0.113*	0.102*	0.101*	-0.037**	0.096**	-0.004**	-0.056**	1.000	
GO	-0.152**	0.297*	-0.146**	-0.057**	0.654*	-0.062*	0.095*	-0.416*	0.135*	-0.053*	-0.454	0.128	1.000

*, **, ***, significant at 10%, 5%, and 1%, respectively.

### 4.3. OLS regression results

Table 4 presents the Ordinary Least Square (OLS) Regression results of Eqs (1) to (3). Before anything else in Model (1), the independent variable green R&D investment is significantly connected to the dependent variables in Model 1 revealing that green R&D investment had a strong connection to corporate GIP (β = 0.0042, P < 0.000). It supports Hypothesis (H1) and is consistent with the study of [135].

**Table 4:** GIP and green R&D investment effects on ESG reporting.

Variables	Model 1 GIP		Model 2 GIP		Model 3 GIP	
GIP	Coefficient	P-Value	Coefficient	p-Value	Coefficient	p-Value
R&D	0.0042 ***	0.000	------------	----------	-0.001	0.002
ESG	------------	----------	0.008***	0.000	0.015	0.000
R&D x ESG	------------	----------	------------	----------	0.009***	0.000
SOEs	-0.003	0.874	0.005	0.817	0.010	0.317
Tobin Q	0.012***	0.000	0.012***	0.000	0.005***	0.001
ROA	0.101***	0.000	0.101***	0.000	0.132***	0.000
FA	-0.000	0.520	-0.000	0.590	-0.000	0.013
FLever	-0.092***	0.000	-0.089***	0.000	-0.084***	0.000
CEOD	0.000	0.821	0.000	0.957	0.0023	0.258
FS	0.005	0.156	0.007	0.754	-0.010	0.324
OC	0.000	0.577	0.001	0.554	0.000	0.976
IO	0.007***	0.003	0.007***	0.002	0.015***	0.000
GO	-0.006	0.030	-0.006	0.028	-0.001	0.246
YI	YES	YES	YES	YES	YES	YES
Constant	0.0318***	0.000	0.035***	0.000	0.050***	0.000
R^2^	0.4244		0.4272		0.4771	

Note

*, **, ***, significant at 10%, 5%, and 1%, respectively.

Secondly, In the second model, the ESG reporting variable is strongly connected to the dependent company GIP. (Table 3) demonstrates that ESG reporting has a favorable influence on GIP (β = 0.008, P < 0.000). Although corporate GIP is included, the company’s ESG reporting remains good. According to the literature [120], We found that Green Innovation does, to some extent, govern the relationship between green R&D investment and ESG reporting, This backs up Hypothesis (H2). According to the findings, green R&D investment can boost company GIP through enhancing ESG reporting.

Lastly, Table 4 model (3) displays the OLS findings of the moderating influence of ESG reporting, corporate GIP, and green R&D investment. As a result, hypothesis (H3) suggests and verifies the link between green R&D spending and GIP with ESG reporting. Furthermore, Model 3 results show a positive and substantial relationship for green R&D x ESG reporting (β = 0.009, p < 0.000) that supports Hypothesis 3, which is consistent with the study of [30, 137].

Furthermore, in Table 4 Model (3), the regression findings of the moderating influence of ESG reporting on the link between GIP and numerous parameters of green R&D investment are presented.

### 4.4. Fixed effects tests results

We used a Fixed Effect test to confirm our main conclusion, which is that corporate GIP is highly connected with ESG reporting and that ESG reporting moderates this relationship [120]. Results suggest that the firm’s GIP can improve the quality of ESG reporting [138]. The value of company green R&D investment was positive and substantial in Model 1, and this green R&D investment coefficient has a favorable influence on corporation GIP (β = 0.004, p < 0.000), In Model 2, ESG reporting moderates the corporate GIP association favorably. Model 2 exhibits a positive coefficient of ESG reporting, indicating that integrating ESG reporting as a moderating factor considerably boosts GIP (β = 0.005, p < 0.000). Overall, our fixed analysis reveals that ESG reporting moderates this association, which is consistent with our primary findings.

Our fixed effect testing is repeated. As far as we know, corporate GIP influences green R&D investment and ESG reporting. These data confirm the concurrent pattern Hypothesis. Table 4 shows that the influence on the interaction term ESG reporting investment is still highly favorable.

Table 5 shows the fixed effects results, which were used to examine the moderating influence and hence decrease potential multicollinearity. ESG reporting, according to hypothesis (3), moderates the combined effect of corporate GIP, green R&D investment, and green R&D x ESG reporting. Model 4 (Table 3) revealed that the interaction term R&D x ESG reporting was connected to corporate GIP in a favorable way (β = 0.008, p< 0.005), demonstrating that ESG reporting mitigates the negative impact of GIP on green R&D investment. Thus, (H3) was supported.

**Table 5:** GIP and green R&D investment impacts on ESG reporting (panel data analysis with fixed effects).

Variables	Model 1 GIP		Model 2 GIP		Model 3 GIP	
GIP	Coefficient	P-Value	Coefficient	p-Value	Coefficient	p-Value
R&D	0.004***	0.000	------------	----------	-0.001***	0.002
ESG	------------	----------	0.005***	0.001	0.021***	0.000
R&D x ESG	------------	----------	------------	----------	0.008***	0.000
SOEs	0.007	0.460	0.008	0.418	-0.005	0.819
Tobin Q	0.005***	0.000	0.005***	0.000	0.013	0.000
ROA	0.133***	0.000	0.133***	0.000	0.098	0.000
FA	-0.005	0.026	-0.000	0.019	-0.000	0.393
FLever	-0.084***	0.000	-0.084***	0.000	-0.099	0.000
CEOD	0.029	0.156	0.002	0.239	0.000	0.921
FS	0.007	0.156	-0.008	0.424	0.007	0.753
OC	0.000	0.569	0.000	0.719	0.001	0.464
IO	0.015***	0.000	0.015***	0.000	0.007	0.002
GO	-0.001	0.025	-0.001	0.222	-0.006	0.019
YI	YES	YES	YES	YES	YES	YES
Constant	0.056***	0.000	0.058***	0.000	0.014 ***	0.000
R^2^	0.4720		0.4714		0.4198	

Note

*, **, ***, significant at 10%, 5%, and 1%, respectively.

### 4.5. Robustness test check

We used two different models to overcome the problem of robustness. A one-year lag model was used by the researcher to re-measure company GIP, green R&D investment, and ESG reporting. Second, A one-year-lagged measure of corporate GIP, green R&D investment, and ESG reporting is used in a two-stage least squares (2SLS) regression (an instrumental variable approach) to solve the robustness problem. Table 6 shows the results of 2SLS regression for Models 1, 2, and 3. Therefore, it is possible to conclude that the results are reliable.

**Table 6:** The influence of GIP, green R&D investment, and the moderating function of ESG reporting (robustness test).

One-year lagged Measure							2-SLS					
Variables	Model 1 GIP		Model 2 GIP		Model 3 GIP		Model 1 GIP		Model 2 GIP		Model 3 GIP	
GIP	Coefficient	P-Value	Coefficient	p-Value	Coefficient	p-Value	Coefficient	p-Value	Coefficient	p-Value	Coefficient	p-Value
R&D	0.005***	0.000	------------	----------	-0.002	0.002	0.002***	0.002	------------	----------	-0.001***	0.003
ESG	------------	----------	0.008***	0.001	0.016	0.002	------------	----------	0.006***	0.004	0.030***	0.001
R&D x ESG	------------	----------	------------	----------	0.009***	0.001	------------	----------	------------	----------	0.009***	0.002
SOEs	-0.004	0.825	0.005	0.886	0.012	0.319	0.007	0.631	0.006	0.604	-0.006	0.812
Tobin Q	0.013***	0.001	0.012***	0.001	0.006***	0.002	0.007***	0.002	0.006***	0.001	0.012	0.001
ROA	0.120***	0.004	0.102***	0.000	0.135***	0.001	0.119***	0.001	0.119***	0.001	0.096	0.001
FA	-0.001	0.562	-0.001	0.598	-0.001	0.014	-0.001	0.078	-0.000	0.065	-0.000	0.350
FLever	-0.080***	0.001	-0.089***	0.001	-0.085***	0.001	-0.082***	0.001	-0.082***	0.001	-0.098***	0.001
CEOD	0.000	0.820	0.001	0.958	0.0024	0.257	0.001	0.224	0.002	0.343	0.001	0.931
FS	0.006	0.154	0.008	0.753	-0.012	0.328	0.006	0.682	-0.005	0.654	0.0072	0.713
OC	0.000	0.578	0.001	0.542	0.0001	0.948	0.001	0.701	0.000	0.609	0.001	0.467
IO	0.008***	0.004	0.008***	0.003	0.016***	0.001	0.013***	0.002	0.012***	0.001	0.008	0.003
GO	-0.007	0.032	-0.007	0.029	-0.001	0.245	-0.002	0.142	-0.002	0.147	-0.008	0.019
YI	YES	YES	YES	YES	YES	YES	YES	YES	YES	YES	YES	YES
Constant	0.0319***	0.000	0.037***	0.000	0.053 ***	0.000	0.058***	0.000	0.058***	0.000	0.054***	0.000
R^2^	0.4246		0.4298		0.4778		0.4197					

Note

*, **, ***, significant at 10%, 5%, and 1%, respectively.

## 5. Discussions and conclusions

Previous research has acknowledged the potential disconnect between investment decisions and their impact on company performance. Our study delves deeper, investigating the role of internal firm mechanisms in bridging this gap, particularly focusing on Environmental, Social, and Governance (ESG) reporting as a moderator influencing the relationship between green Research and Development (R&D) and Corporate Green Innovation Performance (GIP).

ESG reporting has gradually established itself as a requirement for all corporate enterprises. The purpose of empirical research is to investigate the impact of ESG reporting on the link between green R&D and corporate GIP in China, a rapidly increasing industrialized nation. According to prior research, there is an increasing emphasis on the positive benefits of ESG reporting on an enterprise’s financial capabilities [32, 137, 139]. The consequences were assumed to extend to non-financial outcomes.

Our empirical analysis provides strong support for all three proposed hypotheses:

- H1: Green R&D investment has a significantly positive association with Corporate Green Innovation Performance (GIP) (Model 1), confirming its critical role in driving sustainable innovation.
- H2: ESG reporting also exhibits a significant positive correlation with GIP (Model 2), highlighting the value of transparency and communication of green efforts in enhancing a company’s image and performance.
- H3: Most importantly, our results reveal a significant moderating effect of ESG reporting on the relationship between green R&D investment and GIP (Model 3). This means that increased ESG reporting strengthens the positive impact of green R&D on GIP, reinforcing the notion that transparent communication amplifies the effectiveness of green investments.

This finding contributes significantly to the ongoing discussion on the complex relationships between green R&D, GIP, and ESG reporting. It supports theoretical frameworks surrounding agency theory, stakeholder engagement, and resource-based approaches in the context of ESG and green innovation. Our work helps solidify the understanding of how transparent reporting acts as a crucial bridge between green investments and their tangible outcomes in improved GIP. Further investigation into the underlying mechanisms of this moderating effect is warranted.

Imagine a company investing heavily in green R&D, like developing eco-friendly technologies. The results, however, don’t meet expectations. Why? Our research suggests it might be due to a missing piece: transparent communication. We found that ESG reporting, which openly reports environmental, social, and governance efforts, acts as a crucial bridge, amplifying the impact of green R&D on a company’s green innovation performance (GIP). Increased volumes of ESG data build trust with stakeholders, attract resources, and foster collaboration, ultimately unlocking the full potential of green investments. It will enhance Legitimacy and trust with stakeholders, leading to greater support for green initiatives and R&D efforts. Transparent reporting may attract additional resources like funding or partnerships, further bolstering green R&D and innovation capabilities. Open communication of green efforts can foster collaboration with research institutions, environmental agencies, and other stakeholders, accelerating the translation of R&D into GIP.

Our findings paint a clear picture: companies seeking to maximize the impact of their green R&D should embrace ESG reporting as a vital tool. Executives can integrate these strategies, innovate manufacturing processes, and consider ESG indices in their decision-making. Governments can promote transparency through monitoring and green funding initiatives, ensuring the legitimacy and effectiveness of ESG reporting. By working together, businesses and governments can create a symphony of sustainable innovation, where green investments resonate with tangible environmental and financial improvements.

In conclusion, our research demonstrates the multifaceted relationship between green R&D, ESG reporting, and GIP. Increased green R&D investment and transparent communication through ESG reporting are essential for companies to achieve sustainable innovation and success. Importantly, our findings highlight the critical role of ESG reporting in amplifying the impact of green R&D, suggesting a synergistic approach to driving corporate green innovation performance.

### 5.1. Limitations and suggestions for future research

The limitations of this study might inform future research. First and foremost, our data support the existence of a positive relationship between corporate GIP and green R&D expenditure, we recognize that there is still a place for future study to build on our findings. e.g., Future work can analyze the structure or platform used to improve efficiency, especially through ESG reporting. Secondly, we simply used the quantity of green R&D investment input to quantify the variable of green R&D investment. Other types of R&D, including R&D personnel and intellectual capital, may influence ESG’s capacity to access capital.

Green R&D expenditure should be measured, we just used the amount of green R&D investment input. Green R&D in other forms, such as R&D employees and intellectual capital, may influence ESG’s capacity to access financial resources.

Thirdly, Companies interfere in community collaboration, particularly in ESG implementation, because of functional limits and the incapacity to undertake ESG assessments. Future research may further explore the relationship based on the specific content and quality of ESG reporting and its nuanced impact on GIP.

Lastly, we exclusively work with Chinese companies, as a result, the research findings may not apply to other nations. In China, ESG reporting is substantially lower, Furthermore, the firm’s GIP setting is not very reasonable. This result varies greatly between developed and underdeveloped countries, this might limit the breadth of our research findings. Future studies should concentrate on organizations in a variety of more developed nations and compare their findings to those of the current investigation. However, the study’s findings need to be studied further, both qualitatively and quantitatively.

## Supporting information

S1 Data (XLSX)
